# A Data-Driven Predictive Machine Learning Model for Efficiently Storing Temperature-Sensitive Medical Products, Such as Vaccines: Case Study: Pharmacies in Rwanda

**DOI:** 10.1155/2021/9990552

**Published:** 2021-05-03

**Authors:** Joseph Habiyaremye, Marco Zennaro, Chomora Mikeka, Emmanuel Masabo, Kayalvizhi Jayavel, Santhi Kumaran

**Affiliations:** ^1^African Center of Excellence in Internet of Things, College of Science and Technology, University of Rwanda, P.O. Box 3900, Kigali, Rwanda; ^2^International Centre of Theoretical Physics, Strada Costiera, 11, Trieste I-34151, Italy; ^3^Science, Technology and Innovation (DSTI), MoE, Government of Malawi, Capital Hill Circle, Private Bag 328, Capital City, Lilongwe 3, Malawi; ^4^Department of Information Technology, School of Computing, SRM Institute of Science and Technology, Chennai 603203, India; ^5^Department of Information Technology, Copperbelt University, Kitwe 21692, Zambia

## Abstract

Temperature control is the key element during medicine storage. Pharmacies sell some medical products which are kept in fridges. The opening and closing of the fridge while taking some medicine makes the outside hot air enter the fridge, which will increase the inner fridge temperature. When the frequency of opening and closing of the fridge is increased, the temperature may go beyond the allowed storage temperature range. In this paper, we are proposing a model with the help of machine learning that will be used in multiple chambers fridges to keep indicating the time remaining for the inner temperature to go beyond the allowed range, and if the time is short, the system will propose to the pharmacist not to open that particular room and proposes a room that has enough time slots (time to reach the upper limit temperature). By using training data got from a thermoelectric cooler-based fridge, we constructed a multiple linear regression model that can predict the required time for a given room to reach the cut-off temperature in case that room is opened. The built model was evaluated using the coefficient of determination *R*^2^ and is found to be 77%, and then it can be used to develop a multiple room smart fridge for efficiently storing highly sensitive medical products.

## 1. Introduction

In Rwanda, medicines and even some types of vaccines are being sold in pharmacies. Medical products are stored based on their storage conditions, such as temperature, light, and humidity [1]. Some medicines are stored at room temperature, freezer, or refrigerator. Vaccines are mainly used to be kept at a temperature between 2 and 8 degrees Celcius [1, 2]. When a client or patient approaches a pharmacy seeking a vaccine or another medical product that is kept in the fridge, someone who is managing the pharmacy will open the fridge to pick the requested product. When the fridge is opened, the outside hot air will enter the fridge, making the inner side of the fridge gains temperature and loses coldness [3, 4]. If the frequency of opening and closing of the fridge increases, the inner temperature might go beyond the acceptable storage range, and this may lead to the inefficacy of the stored medical products [4].

In this work, we propose a predictive model that can be embedded in a fridge with multiple chambers to keep displaying the remaining time slot for every chamber to reach the cut-off temperature (the upper-temperature range). In this work, we assume that the fridge contains only products with identical storage conditions. This model uses the historical data about how long it takes for the temperature to go beyond the acceptable range when the fridge is opened, the initial inner temperature of the fridge at the time of opening, the outside temperature at the opening time, and the time of the day at which the fridge got opened. To get training data for our model, we have developed a fridge using Peltier cooler kits, a microcontroller, temperature sensors, and magnetic switches. Data generated from the fridge were sent to a remote database through GPRS protocol. We have randomly opened the fridge simulating the way the fridge is being opened while picking medicines in pharmacies, but that time we opened the fridge and waited for the inner temperature to rise and reach the maximum allowed storage temperature for the medicine under consideration, then we recorded the initial opening temperature (the temperature at opening time), the outside temperature, the time taken for the temperature to reach the maximum allowed temperature, and the time of the day at which the fridge got opened.

Data were manually fetched from the database and then used for model training and other analysis.

Our contribution was to propose a machine learning model which is based on linear regression with multiple variables that can be embedded in a fridge (multichambers fridge) to make it enough intelligent for monitoring the opening and closing of the door for proper storage of temperature-sensitive products such as vaccines.

## 2. Related Works

The idea of intelligent refrigerators is not new. This section summarizes some works related to smart fridges. A lot of researchers proposed fridges that can be remotely monitored with the help of the Internet of things, a fridge that can help in monitoring the expiration date of refrigerated products, and others proposed fridges that can help in the management of food wastage. Livingston et al. and the team [5] proposed a smart home fridge (that keeps vaccines) which is programmed in the way that it will keep monitoring the action of opening and closing of the door to check if the patient is regularly taking medicines, considering that he/she is taking medicine at regularly known intervals of time. If the fridge is not opened at the corresponding time, it will send some notification to the doctor or a family member. The article at [6] details an IoT-based fridge where it can be seen from a remote area if vaccines are stored at the right temperature. The article in [7] talks about an intelligent fridge that gives alerts when there was a power failure, fridge failure, or even when the door was left open. Weka Solutions [8] developed an IoT platform (Azure IoT Platform) that collects data from sensors from the vaccine fridge in a real-time manner and this fridge is working on Raspberry Pi 2. Works in [9, 10] proposed a smart fridge from which it is possible to get information about products remaining inside and it is possible to know the status of its door with the help of RFID technology. The research work in [11] proposes a medical fridge to improve the healthcare system by using the barcode reader system. The system scans the barcode for each medicine to keep tracking the expiration date. It also has a camera to keep monitoring the fridge content and this can be done from remote locations. Articles in [12–16] worked on a refrigerator that is based on IoT for remotely monitoring for different parameters in real-time mode. Articles in [17–19] proposed different methods related to the smart refrigerator for avoiding food wastage in a fridge. When it comes to remote control or monitoring of patient-related items through the Internet, security has to be taken under consideration even if it is not directly related to the current work, but we have decided to incorporate the security aspect as part of our future works. In the following works, the authors elaborated on different important security aspects that can be used in IoT systems. The work in [20] proposed security aspects that can be considered in the term of the Internet of Medical Things (IoMT); this can be used in our medical fridge too. In the article [21], a blockchain-based security mechanism is explained, though the application is used for verification in a smart city context. This also serves as an inspiration to add security aspects to our medical fridge in terms of blockchain-enabled technology. The work in [22] discussed the concept of a Cache Distributed System, with the help of two servers, one Cloud server, and an Edge Server. This emphasizes the importance of incorporating 6G in cases that involve big data. This can also be applied in our case as well. On the fridge side, some authentification can also be added so that it could be accessed by only individuals for better and safer handling. The work in [23] gives some details on how security can be achieved by fingerprint images with an optimal compression ratio.

To the best of our knowledge, this the only research work that proposes a machine learning model to be embedded in a medical multichambers fridge to help pharmacists to achieve an efficient way of storing medical products by predicting the remaining time for a particular chamber to go beyond the accepted storage temperature.

## 3. Proposed Model

To efficiently manage the storage of medicines, especially temperature-sensitive products, such as vaccines. We propose a multiple chamber fridge with an embedded controller that can run a predictive machine learning model [24]. The proposed model is shown in Figure 1 and works based on the flowchart of Figure 2.

From the above figure, the proposed fridge has multiple rooms (four in our case). Each room has an inside temperature sensor to keep monitoring the temperature, a door magnetic sensor to get information about the door condition (closed or opened), and an outside temperature sensor (common for all rooms). The fridge also has a screen from where a user can see different room conditions including the current room temperature, the room door status, and the time remaining for each room to get the cut-off temperature (the maximum allowed temperature). Apart from that, the fridge has a GSM modem that is transmitting data to a remote database for remote monitoring or for saving data for further research.

From our experiments, we found that the time to cut-off temperature depends on the following:

- The initial room temperature (the temperature at the opening time). If this temperature is high (approaching the cut-off temperature), the time to cut-off temperature will be short.
- The time of the day. Particularly, in Rwanda, the temperature will increase with time, especially when we have a sunny day. During morning time, it is somehow cold and the temperature rises by the time and starts reducing by evening time. This temperature change will have some impact on the inner fridge temperature due to heat transfer through fridge walls.
- The outside air temperature.

In addition to the above parameters, it is clear that this time slot depends even on the angle at which the fridge is being opened and the outside atmospheric pressure. However, in our experiments, we have ignored the impact of atmospheric pressure, and we have kept the opening angle constant.

We propose that when the pharmacist wants to pick a vaccine, he/she will first take a look at the display to check for which room has a long time. If the time to cut off temperature is found to be short, the pharmacist can even wait for some time. The process can be explained with the flowchart of Figure 2.

## 4. Materials and Methods

During our research work, we tried to generate data to be used for model training. The following section gives all details about how we got the data that have been used.

### 4.1. Single Room Fridge Development

To generate data, we built a four-chamber fridge (undergoing research), Figure 3, and from this fridge, we did our study on one of the chambers of this fridge (the main chamber).

The cooling system for this fridge is made of thermoelectric coolers [25, 26]. Each of the four rooms in our fridge has an inside temperature sensor and a door magnetic switch to know if a particular room is open or closed. Apart from this, there is an outside temperature sensor to get information about the outside environment temperature. The details about the fridge construction are shown in Figure 4.

### 4.2. Fridge Components

To generate data to be used for model training, an electronically controlled fridge that is made from thermoelectric technology was developed. The fridge has two main components:

#### 4.2.1. Thermoelectric Cooler System

This is the part that generates cooling. It is made of a combination of two fans, a heat sink, and a TEC device. In short, when a TEC device is supplied by a DC voltage, one side will be hot while another one will be cold [27]. To bring the generated low temperature to our room/chamber, we used one fan and another fan was used to take out the generated high temperature. The cooling room is made up of two TEC kits, one on the left side while another on the right side. Details can be seen in Figure 5.

#### 4.2.2. Controller and Radio Unit

The cooling system (TEC Systems) and fridge systems are controlled by Arduino Mega (Arduino, Turin, Italy) through temperature and door magnetic sensors.

The radio unit is made by a SIM800L (SimCom, Shangai, China) which is transmitting data to a remote database through GPRS protocol from where data are manually downloaded in CSV format for model training purposes. The controller was programmed to read sensors (temperature and door magnetic switch) and count the time passed when a particular door is opened and finally send this data to the GSM modem.

### 4.3. Data Generation

As our target was to know the impact of opening and closing of the fridge while picking some medicines, the data generated from this fridge were sent to a remote database for storage as this was our easiest method of saving data. This paper is a small portion of the other research work which is under progress where we monitor and control a four-chamber fridge with the help of the Internet of Things. However, in this work, we only work with data from a single room; Figure 6 gives details on how data are generated and transmitted to the remote database.

We tried to simulate the process of opening and closing the medical fridge by the pharmacist while picking medicines.

The constructed fridge was able to reduce the fridge room temperature up to 9 Celcius degrees.

To achieve our simulation, we considered a temperature range of 10–18 degrees (we could take a normal vaccine range (2–8 Celcius degree); however, our cooling system could not help) and used it to randomly open and wait for the chamber temperature to hit up range (18 Celcius degrees), if the upper acceptable temperature is reached, the buzzer used to ring. We used to close the door and wait for some random time and repeat the operation.  Figure 7 shows the flowchart that indicates the way we generated data.

Generally, we send the status of the door (open or closed), the chamber temperature, the outside temperature, how long the chamber has been opened (in the case it is opened), and the time stamp.

### 4.4. Model Training

To find a relationship between independent variables (outside temperature, inside chamber temperature, and the time of the day) and the dependent variables (the time to be taken to reach the upper acceptable temperature), we used linear regression with multiple variables, also known as multivariate regression [28].  Figure 8 shows the relationship between different parameters used in our model: The outside temperature (OuTemp), inside temperature (InTemp), the time day (Day_Time), and the time during which the fridge has been opened for reaching the cut-off temperature (Time_Opened_Min).

The inside temperature, outside temperature, and daytime are taken as independent variables, and the time required for the room temperature to reach the cut-off temperature is taken as the dependent variable. Variables are explained in Table 1 and the statistics details of the variables are shown in Table 2.

The linear regression with multiples features equation can be written as follows:

(1) $$\begin{array}{c} T_{\text{cut}-\text{off}}=m_{1}*\text{OuTemp}+m_{2}*\text{InTemp}+m_{3}*\text{DayTime}+\beta , \end{array}$$

where *T*_cut−off_ is the time required for the room temperature to hit the upper-temperature range, OuTemp is the outside temperature, InTemp is the inside temperature, DayTime is the daytime, *m*_*n*_ is the coefficient, *β* is the intercept.

### 4.5. Data Preprocessing

While sending data to a remote server, the server was used to provide a timestamp in HH:MM: SS XM format means a 12H system. To easily use a timestamp in our model, we converted it to HH:MM: SS means a 24 H system. Our target was to count a day from the 1^st^ hour to the 24^th^ hour and considering that hours of a day can impact the model differently. Tables 3 and 4 indicate only ten rows of our dataset. Apart from the timestamp, the period in which the fridge got opened has been considered in minutes. Details about how the data have been converted before being used for model training are shown in Tables 3 and 4.

## 5. Results and Discussion

During our experiment, we recorded the data for 3 months. However, we simulated the selling process for 12 days. Figures 9 and 10 give details about the different results. From these figures, we can easily see that the process of opening and closing a fridge has a big impact on the chamber temperature. From Figure 10(a), we see that the selling process happened only during the daytime and it is also seen that during the daytime, the temperature (for both inside and outside) increases while the temperature reduces during nighttime. This explains that the daytime has an impact on the temperature too.

The above details show that the fridge's inside temperature varies when the fridge is being opened. From the same graphs, we can also see that the outside temperature will vary based on the time of the day. During the daytime, even if the door is closed, we can observe some increase in inside temperature which is due to heat exchange between the outside medium and the inside medium.

It can be seen that the fridge room temperature depends on how frequently is being opened, the time of the day, and the outside temperature. And the period for the inside temperature to reach the upper-temperature limit depends on the initial temperature at the opening time, the time of the day and, the outside temperature.

### 5.1. Model Results and Prediction Accuracy

In this section, we have different results which show that our model is accurate.  Figure 11 indicates how each predictor variable is related to the target variable.

From the above figure, we can conclude that the chamber temperature and the outside temperature have more contribution to the model than the daytime.

Table 5 shows some numerical results for checking the accuracy of our model. From this table, we can see that the coefficient of determination is equal to 0.767. Thus, the model is not less effective and efficient. Looking at results from Figure 12 of residuals plots), points are randomly dispersed around the *x*-axis. This indicates that heteroscedasticity is not an issue with predictor variables [29–31]. Then our model is appropriate and the results from the analysis can be taken as valid.

From the above Table 6,

*m*_1_ = −0.58, *m*_2_ = −0.53, *m*_3_ = 0.0016, *β* = 23.4.

Then equation (1) can be rewritten as follows:

(2) $$\begin{array}{c} T_{\text{cut}-\text{off}}=-0.58*\text{OuTemp}-0.53*\text{InTemp}+0.0016\text{DayTime}+23.4. \end{array}$$

Considering the above coefficient of Table 5 and model results, we can say that

- When the outside temperature increases, it will take a short period for the inside temperature to reach the cut-off temperature.
- It is even the same for the inside temperature (at the opening time). If it is higher, it will also take a short period to reach the cut-off temperature.
- Considering the *P*values of dependent variables, the inside temperature and the outside temperature contribute more to the prediction comparing to the daytime.

During our research work, we initially considered a deep Neural Network algorithm, but in the end, we found that the regression model works better than the Neural Network.  Table 7 summarizes the results from the two algorithms.

## 6. Conclusions

In this work, a machine learning method to predict the remaining period for the temperature inside a fridge to go beyond the acceptable range has been developed. The developed model has to be embedded in the fridge that has a controller with enough resources to run a machine learning model. The proposed model will keep monitoring the impact of opening and closing of the fridge while picking some products.

Results from our analysis show that the model was accurate at 0.77, which means that 77% of the total variation in time to cut-off temperature is explained by the regression. *P* values for both the inside temperature and outside temperature are below 0.05, and then it can be concluded that those two parameters have considerable contributions on the prediction of the time required for the chamber temperature to reach the upper acceptable range.

The experiment showed that when the outside temperature increases by one degree Celcius, the time to cut-off temperature is reduced by 0.58 minutes. When the inside temperature is kept constant and when the chamber temperature increases by one degree Celcius, the time to cut-off temperature is reduced by 0.53 minutes when the outside temperature is kept constant.

The proposed model is useful for pharmacies that sell medical products (case of Rwanda). We also proposed that to efficiently store temperature-sensitive medical products, the proposed model has to be used in a multiple chambers fridge with a screen from where the remaining period for cut-off temperature will be displayed. In this case, someone in charge, before opening the fridge, will check and open the chamber that indicates a longer period. The Internet of Things can also be integrated into the proposed solution for remote monitoring and control purposes.

## Figures and Tables

**Figure 1:** Proposed fridge.

**Figure 2:** Proposed model flow chart.

**Figure 3:** Four-chamber fridge.

**Figure 4:** Data generation system diagram.

**Figure 5:** Fridge components & data generation details.

**Figure 6:** Data generation process.

**Figure 7:** Training mode data generation flow chart.

**Figure 8:** Relationship between variables under consideration.

**Figure 9:** Experimental results. (a) The outside temperature variation due to climate, (b) The inside temperature variation due to opening and closing. (c) Opening and Closing (closed = 1, open = 0). (d): Consolidated graph.

**Figure 10:** One-day simulation results. (a) Analysis of the whole day results. (b) analysis during a portion of time ∼ two hours.

**Figure 11:** The contribution of independent variables. (a) The relationship between the dependent variable and the chamber temperature. (b) The relationship between the dependent variable and the outside temperature. (c) The relationship between the dependent variable and the daytime.

**Figure 12:** Model residuals analysis. (a): residuals versus the chamber temperature. (b): residuals versus the outside temperature. (c): residuals versus the daytime.

**Table 1:** Explanatory variables considered in the regression model to predict the time to cut-off temperature.

Variables	Description	Units
OuTemp	The outside temperature at opening time	°C
InTemp	The inside room temperature at opening time	°C
DayTime	The day time at the time of fridge opening	Hours

**Table 2:** Descriptive statistics of independent variables.

Independent variables	TempOut (°C)	InTemp (°C)	Day_hour
Mean	22.4	14.9	12.24
Std	0.79	1.52	3.24
Min	20.56	11.63	7.2
Max	24.8	17.81	17.8

**Table 3:** Initial data: before preprocessing.

OuTemp (°C)	InTemp (°C)	Time_open (sec)	Time_stamp
22.25	14.75	136	8:39:10
22.31	13.69	168	8:54:45
22.31	15.56	95	9:03:33
22.37	14.81	144	9:14:32
22.37	17.37	71	9:19:08
22.44	17.81	22	9:21:19
22.44	15.88	95	9:27:00
22.44	17.19	54	9:31:28
22.44	17.37	38	9:35:16
23.19	15.44	95	1:41:38

**Table 4:** Final data. After preprocessing.

OuTemp [°C]	InTemp (°C)	Time_open (sec)	Time_open (min)	Time (12 H)	Time (24 H)	Day_hour
22.25	14.75	136	2.3	8:39:10	8:39:10	8.7
22.31	13.69	168	2.8	8:54:45	8:54:45	8.9
22.31	15.56	95	1.6	9:03:33	9:03:33	9.1
22.37	14.81	144	2.4	9:14:32	9:14:32	9.2
22.37	17.37	71	1.2	9:19:08	9:19:08	9.3
22.44	17.81	22	0.4	9:21:19	9:21:19	9.4
22.44	15.88	95	1.6	9:27:00	9:27:00	9.5
22.44	17.19	54	0.9	9:31:28	9:31:28	9.5
22.44	17.37	38	0.6	9:35:16	9:35:16	9.6
23.19	15.44	95	1.6	1:41:38	13:41:38	13.7

**Table 5:** Regression model results.

	Coef	Std err	*T*	*P* > |*t*|
Intercept	23.405	1.199	19.520	0.000
InTemp	−0.5328	0.027	−20.093	0.000
OuTemp	−0.5838	0.055	−10.558	0.000
Day_Hour	0.0016	0.014	0.120	0.905

**Table 6:** More about regression model results.

Parameter	Value
*R*-squared	0.767
Adj. *R*-squared	0.763
*F*-statistic	195.2
Prob (*F*-statistic)	4.90*e *−* *56
Log-likelihood	−142.47
AIC	292.9
BIC	305.8

**Table 7:** Comparison between neural network and linear regression on our datasets.

True value [Min]	Predicted_linear_reg	Predicted_DNN
2.3	2.5	2.6
2.8	3.1	3.1
1.6	2.1	2.0
2.4	2.4	2.4
1.2	1.1	2.0
0.4	0.8	2.0
1.6	1.8	1.9
0.9	1.1	2.0
0.6	1.0	2.0
1.6	1.6	2.1
1.1	0.9	2.0
3	2.8	2.5
1.3	1.1	2.1
4.2	3.2	2.3
3.5	3.2	2.4
4.3	3.2	2.7
3.2	3.2	2.9

Column 2 of Table 7 (the linear regression predicted values) can even be verified using equation (2).

## Data Availability

The data used to support the findings of this study are available from the corresponding author upon request.
